# DDTC Suppresses Ovarian Cancer Development via the PI3K/AKT/mTOR Signaling Pathway

**DOI:** 10.1155/2022/1941077

**Published:** 2022-08-08

**Authors:** Meng Li, Wenqi Zhang, Yihan Wang, Kai Huang, Tao Sun, Zhicong Qiu, Linqi Yang, Meng Wu, Xiaolu Zhang, Wei Zhang

**Affiliations:** ^1^Department of Pharmacology, College of Basic Medicine, Hebei University of Chinese Medicine, Shijiazhuang, 050200 Hebei Province, China; ^2^Department of Hematology, The Fourth Hospital of Hebei Medical University, Shijiazhuang, 050000 Hebei Province, China; ^3^Department of Gastroenterology, Qinhuangdao Beidaihe Hospital, Qinhuangdao, 066199 Hebei Province, China

## Abstract

In prior research, 6,12-diphenyl-3,9-diazatetraasterane-1, 5, 7, 11-tetracarboxylate (DDTC) has been shown to be an effective inhibitor of the growth of the SKOV3 and A2780 ovarian cancer (OC) cell lines. Flow cytometry analyses indicated that DDTC was able to suppress P-CNA expression at the protein level within OC cells, while RNA-seq indicated that DDTC treatment was associated with marked changes in gene expression profiles within A2780 cells. Molecular docking analyses suggested that DDTC has the potential to readily dock with key signaling proteins including PI3K, AKT, and mTOR. In line with these findings, DDTC treatment inhibited the growth of xenograft tumors in a mouse model system. Such treatment was also associated with reduced p-PI3K/PI3K, p-AKT/AKT, p-mTOR/mTOR, and CyclinD1 (CCND1) expressions and with the increased expression of PTEN *in vitro* and *in vivo*. Together, these results suggest that DDTC is capable of readily inhibiting OC development at least in part via targeting and modulating signaling via the PI3K/AKT/mTOR axis.

## 1. Introduction

Ovarian cancer (OC) is the deadliest and second most common form of gynecological malignancy, with advanced OC patients exhibiting a 5-year survival rate of just 30% [1]. Surgical tumor resection, chemotherapy, and radiotherapy are the mainstays of OC treatment [2, 3]. However, the chemotherapeutic agents most commonly used to treat this cancer type (cisplatin, paclitaxel, and cyclophosphamide) are associated with high rates of drug resistance and adverse reactions. There is thus a clear need for the discovery or development of novel antitumor medications capable of safely and effectively treating OC.

The development of effective, novel, natural therapeutic approaches to OC tumor-targeting remains limited. DDTC was synthesized as a protease inhibitor capable of interfering with human immunodeficiency virus- (HIV-) 1 replication [4, 5]. DDTC has also been shown to exhibit robust antitumor activity, highlighting its potential as a therapeutic agent in patients with OC [6]. The mechanisms whereby DDTC may modulate OC tumor cell growth, however, have yet to be characterized. In this study, we thus explored the mechanistic role of DDTC as a regulator of the *in vitro* and *in vivo* apoptotic death of OC cells.

## 2. Materials and Methods

### 2.1. Main Drugs and Reagents

Fetal bovine serum (FBS) was obtained from Hyclone (USA), while RPMI-1640, penicillin/streptomycin, and all other reagents were from GIBCO (USA). DDTC was synthesized by the College of Chemical Engineering, Shijiazhuang University, and dissolved in PEG-400 prior to storage at 4°C.

### 2.2. Cell Culture

RPMI-1640 containing 10% FBS and penicillin/streptomycin was used to culture the human SKOV3 and A2780 OC cell lines in a humidified 37°C 5% CO_2_ incubator.

### 2.3. Flow Cytometry

Initially, a range of DDTC concentrations (0.1, 1, and 10 *μ*M) were used to treat SKOV3 and A2780 cells for 48 h, after which cells were harvested with trypsin and stained with AF488-conjugated anti-human PCNA at 4°C. Cells were then analyzed with a FACSCalibur system (BD Biosciences, NJ, USA).

### 2.4. RNA-seq

RNA-sequencing (RNA-seq) was conducted to explore the effects of DDTC treatment on OC cell transcriptomic profiles (*n* = 2). TRIzol (Invitrogen, CA, USA) was used to isolate RNA from A2780 cells treated with or without 1 *μ*M DDTC in triplicate (RNA concentrations: 23.8-41 ng/*μ*L. The integrity of isolated RNA was assessed with Agilent Bioanalyzer 2100 (Agilent Technologies, CA, USA), yielding RIN values of approximately 9.4. A VAHTS Stranded mRNA-seq Library Prep Kit for Illumina® (Vazyme Biotech, Nanjing, China) was used for paired-end library preparation based on provided directions. All library construction and sequencing were conducted by Shanghai Biotechnology Corporation (China). Significantly expressed genes (SEGs) were identified using the following criteria: false discovery rate (FDR) < 0.05 and fold change ≥ 2. Differentially expressed genes (DEGs) were then subjected to GO (http://www.geneontology.org/) and KEGG pathway enrichment analyses.

### 2.5. Molecular Docking

PI3K pathway signaling proteins were selected to conduct molecular docking analyses. The protein database (http://www.pdb.org/) was used to download crystal structures for PI3K (PDB ID:1E8W), AKT (PDB ID:3O69), and mTOR (PDB ID:2FAP). DDTC was drawn with ChemDraw 18.0. AutoDock Vina was used for molecular docking and conformation scoring, with optimal docking result structures then being drawn with PyMOL and Maestro 11.9.

### 2.6. Relationship between the mRNA Levels of Related Genes and the Survival Outcomes of Patients with OC

We utilized R3.6.3 software to carry out the receiver operating characteristic curve (ROC curve) and the Kaplan-Meier curve (KM curve) enrichment analyses. We prepared RNA-seq data and clinical p from ovarian serous cystadenocarcinoma (OV) project in TCGA (https://portal.gdc.cancer.gov/), transformed them into transcripts per million reads (TPM) format, and then analyzed them according to the molecular expression.

### 2.7. Xenograft Ovarian Tumor Mouse Models

Female BALB/C nude mice (6-8 weeks old; 20-25 g) were obtained from Beijing Vital River Laboratory Animal Technology Co., Ltd. (China) and housed under specific pathogen-free conditions within laminar flow cabinets. The Institutional Animal Care and Use Committee of Hebei Medical University approved all animal research (approval ID: SYXK2018-005).

To establish tumors, cells in the logarithmic phase of growth were harvested, rinsed twice using RPMI-1640, and suspended in sterile PBS. The right foreleg of each mouse was then subcutaneously implanted with 0.2 mL of tumor cells (2 × 10^6^/mL). Mice were then randomized into A2780-PEG-400 and A2780-DDTC groups (*n* = 6/group), with mice in A2780-PEG-400 and A2780-DDTC groups receiving subcutaneous injection of 0.333 mM PEG-400 (in 2 mL) and 0.333 mM DDTC (in 2 mL) every other day, respectively. Tumor volumes and body weight were recorded every day. Tumor volume was measured as follows: *V* = (*a* × *b*^2^)/2 (cm^3^), with *a* and *b*, respectively, corresponding to the height and width of the tumor. After 14 days, tumors were harvested, weighed, snap-frozen, and transferred to -80°C.

### 2.8. qRT-PCR

TRIzol was used to collect RNA from cells in different treatment groups as above based on provided directions, with spectrophotometric analysis at 260 nm being used to assess RNA purity and concentrations. A PrimeScript RT Reagent Kit (Takara Co., Ltd., USA) was used to prepare cDNA from 1 *μ*g of total RNA, after which qRT-PCR was conducted with a Real-Time PCR System (Bio-Rad Co., Ltd., USA) in a 25 *μ*L volume containing cDNA, primers (Table 1), and TB Green Premix Ex Taq II (Takara Co., Ltd., USA).

### 2.9. Western Blotting

After rinsing cells and tissue samples three times using PBS, they were lysed on ice for 30 min and spun down for 5 min at 10,000 × *g* at 4°C. Protein concentrations were measured using a ND-1000 Spectrophotometer (NanoDrop, DE, USA). Equal protein concentrations were then separated via 10% SDS-PAGE and transferred onto PVDF membranes (Millipore, MA, USA). Blots were then blocked using 5% BSA for 2 h, probed overnight with primary antibodies specific for p-AKT (GB13012-3, 1 : 500), AKT (GTX28805, 1 : 800), p-PI3K (GTX132597, 1 : 800), PI3K (ab40755, 1 : 1000), p-mTOR (ARG51712, 1 : 800), mTOR (GTX101557, 1 : 800), PTEN (ET1606-43, 1 : 800), CyclinD1 (ab134175, 1 : 1000), and *β*-actin (AC026, 1 : 10000) at 4°C, and incubated with secondary goat anti-rabbit IgG (KPL074-1506, 1 : 5000) for 1 h at 37°C. A Fusion FX5 Spectra (Fusion, France) approach was then used to detect protein bands and to assess their density.

### 2.10. Statistical Analysis

Data are means ± standard deviation (SD) from multiple experimental replicates. Data were compared via one-way ANOVAs with the S-N-K test, and the significance threshold was *P* < 0.05.

## 3. Results

### 3.1. DDTC Treatment Modulates Multiple Cancer-Related Pathways within OC Cells

To explore the mechanisms whereby DDTC can impact tumorigenic processes in OC cells, an RNA-seq analysis of A2780 cells that had been treated with or without DDTC was initially performed. In total, 2310 DEGs were identified via this approach, of which 724 and 1586 were, respectively, upregulated and downregulated in DDTC-treated cells relative to control. GO and KEGG analyses of these genes revealed DDTC to impact key cancer-associated pathways including the cell cycle, TGF*β*, cGMP-PKG, and PI3K signaling pathways (Figure 1).

### 3.2. Molecular Docking Analyses

Next, AutoDock Vina was used to conduct molecular docking simulations exploring potential interactions between DDTC and different PI3K signaling pathway proteins; all three tested proteins exhibited good binding energy values (−7.4 to −9.0 Kcal/mol) for DDTC. Moreover, DDTC was found to form hydrogen bonds with GLY945, ARG982, and TYR1050 residues in PI3K, with ARG982 forming a hydrophobic interaction. In addition, DDTC was predicted to engage in hydrophobic interactions with PRO388, LYS389, PRO42, and TYR38 residues in AKT, in addition to hydrogen bonding with VAL45 at the AKT binding site. Similarly, DDTC was predicted to engage in hydrogen bonding with the GLU54, ASP2102, and THR2098 residues of mTOR, with hydrophobic interactions with PHE46, TYR26, PHE2039, TYR2105, and PHE2108, and with electrostatic interactions with the mTOR GLU54 residue (Figure 2).

### 3.3. Relationship between the mRNA Levels of Related Genes and the Survival Outcomes of Patients with OC

We further explored the critical efficiency of related genes in the survival of patients with OC. The ROC curve analysis for PI3K, AKT1, mTOR, PTEN, and CCND1 in OC determined that AUC of the ROC curves is more than 0.640. The Kaplan-Meier curve and log-rank test analysis revealed that variation in AKT1, mTOR, PTEN, and CCND1 mRNA levels was significantly associated with the overall survival (OS) of OC patients (Figure 3).

### 3.4. The Impact of DDTC on Cell Proliferation Progression

A CCK-8 assay suggested that DDTC treatment is associated with antiproliferative activity. Flow cytometry analyses further indicated that 10 *μ*M DDTC treatment suppressed P-CNA expression within both A2780 and SKOV3 cells (Figure 4), suggesting that DDTC can suppress the proliferation of cells.

### 3.5. DDTC Treatment Inhibits the *In Vivo* Growth of OC Tumors

To explore the functional value of DDTC as a regulator of tumorigenesis, the impact of such treatment on the growth of A2780 tumor xenograft growth in nude mice was assessed. Significantly slower tumor growth was observed following DDTC treatment relative to control treatment, confirming the *in vivo* antitumor potential of this therapeutic drug (Figure 5).

### 3.6. DDTC Suppresses the *In Vitro* and *In Vivo* Expression of PI3K-AKT Pathway

Next, qRT-PCR analyses were conducted revealing significant reductions in PI3K, AKT, mTOR, and PTEN mRNA levels in response to DDTC treatment (*P* < 0.05), with the same also being evident in xenograft tumors harvested from mice (Figure 6). Similarly, p-PI3K/PI3K, p-AKT/AKT, p-mTOR/mTOR, and CCND1 were downregulated at the protein level in DDTC-treated groups both *in vitro* and *in vivo*, while PTEN was upregulated (Figure 6). These results suggest that DDTC treatment is capable of effectively inhibiting the activation of the PI3K-AKT signaling pathway in OC cell lines and xenografts.

## 4. Discussion

In prior reports, DDTC has been shown to inhibit the migratory, invasive, and cell cycle progression activity of OC cells [6]. Similarly, the results of the present study support the marked antitumor efficacy of DDTC treatment against OC *in vitro* and in murine xenograft models.

The acidic nucleic acid protein proliferating cell nuclear antigen (P-CNA) is a critical DNA synthesis-related polypeptide that can be analyzed to gauge cellular proliferation, with altered P-CNA expression corresponding to a change in cell proliferation progression. It can specifically reflect the state of cell proliferation. As such, analyses of PCNA can offer an efficient means of gauging the proliferative status of tumor cells. High levels of P-CNA expression have been reported in OC and in other cancers such as gastric, lung, liver, and breast cancers [7, 8]. Notably, DDTC treatment inhibited P-CNA expression by OC cells in vitro in the present analysis. Further RNA-seq studies indicated that DDTC is capable of modulating several key tumor-associated molecular pathways including the cell cycle, TGF*β*, cGMP-PKG, and PI3K signaling pathways. In particular, the PI3K signaling pathway was identified as an important treatment-related target in GO and KEGG enrichment analyses. Consistent with this finding, molecular docking analyses suggested that DDTC is capable of readily interacting with key protein components of this signaling pathway including PI3K, AKT1, and mTOR.

In prior clinical studies, up to 70% of OC cases were found to exhibit PI3K/AKT pathway dysregulation related to PIK3CA mutations and PTEN deletions [9]. Changes in AKT pathway activity can alter tumor cell migratory, invasion, and autophagic activity, making this pathway a promising target for therapeutic intervention in OC [9–12], with several PI3K/AKT/mTOR pathway inhibitors having shown promise in the OC treatment in the clinic [9]. PTEN is a primary negative regulator of the PI3K/AKT pathway, which regulates the cell division cycle by preventing cell growth and unregulated division. PTEN can modify other proteins and lipids through dephosphorylation. PTEN sends signals to cells to stop division and proceed to apoptosis, thus reducing tumor growth [13, 14]. CCND1 has been recognized as a oncogene, and overexpression of CCND1 can lead to uncontrolled cell proliferation. Studies have shown that overexpression of the CCND1 has been identified in various cancers, including breast cancer, bladder cancer, and lung cancer [15, 16].

In the light of the above evidence, the PI3K pathway may represent a core component of the signaling machinery targeted by DDTC treatment in OC. In this study, qRT-PCR and Western blotting were used to explore the mechanisms whereby DDTC induces tumor cell apoptosis. Following DDTC treatment, SKOV3 and A2780 cells exhibited decreased PI3K, AKT, mTOR, and CCND1 mRNA levels as well as reduced p-PI3K/PI3K, p-AKT/AKT, p-mTOR/mTOR, and CCND1 protein levels and increased the expression of PTEN, suggesting that DDTC can drive apoptotic death via the inhibition of the PI3K/AKT/mTOR signaling pathway.

## 5. Conclusion

In conclusion, the results of this study demonstrated that DDTC is capable of inhibiting the PI3K/AKT/mTOR signaling activity within OC cells *in vitro* and in xenograft models, suggesting that this drug may be capable of inducing tumor cell apoptosis in part through this pathway. As such, OC holds great promise as a drug suitable for treating patients with OC.

## Figures and Tables

**Figure 1:** RNA-seq analyses of A2780 OC cell transcriptomic changes in response to DDTC treatment. GO (a) and KEGG pathway (b and c) enrichment analyses of DEGs identified when comparing A2780 cells treated with DDTC and control analyses.

**Figure 2:** Molecular docking results. Interactions between PI3K (a), AKT1 (b), mTOR (c) protein, and DDTC (3D). (d) DDTC structural diagram.

**Figure 3:** Relationship between the mRNA levels of related genes and the survival outcomes of patients with OC. (a) The ROC curve of related genes in OC. (b) The expression of related genes differs in OC. ^∗∗∗^*P* < 0.001. (c–f) The KM curve of related genes in OC.

**Figure 4:** Flow cytometry analyses of protein expression by flow cytometry. SKOV3 and A2780 cells were treated with DDTC (0.1 *μ*M, 1 *μ*M, and 10 *μ*M), resulting in reduced P-CNA protein expression. ^∗^*P* < 0.05.

**Figure 5:** The impact of DDTC treatment on A2780 xenograft tumor growth *in vivo*. (a) Schedule of tumor implantation and injection of PEG-400 or DDTC for cell depletion in mice. (b) Xenograft tumor volume was monitored over time in the two treatment groups. Tumors were weighed in the PEG-400 and DDTC groups. (c and d) DDTC treatment suppressed A2780 xenograft tumor growth following implantation into nude mice (*n* = 6). ^∗∗^*P* < 0.01.

**Figure 6:** (a and b) Western blotting revealed reductions in p-PI3K, p-AKT, p-mTOR, and CCND1 protein levels and increased PI3K, Akt, mTOR, and PTEN protein levels following the DDTC treatment of A2780 cells. (c) qRT-PCR was used to examine the effect of DDTC treatment on PI3K-AKT pathway-related gene expression within A2780 cells. (d and e) Western blotting revealed reductions in p-PI3K, p-AKT, p-mTOR, and CCND1 protein levels as well as increases in PI3K, AKT, mTOR, and PTEN protein levels in SKOV3 cells following DDTC treatment. (f) qRT-PCR was used to examine the effect of DDTC treatment on PI3K-AKT pathway-related gene expression within SKOV3 cells. (g–i) Western blot and qRT-PCR indicated that p-PI3K/PI3K, p-AKT/AKT, p-mTOR/mTOR, and CCND1 were significantly downregulated and PTEN was upregulated at the mRNA and protein levels in A2780 cell-derived tumor xenografts following DDTC treatment relative to control PEG-400 treatment. ^∗^*P* < 0.05 and ^∗∗^*P* < 0.01 vs. control group. OC cells were treated with a range of DDTC doses (0.1, 1, and 10 *μ*M).

**Table 1:** qRT-PCR primers.

Primers	Forward (5′-3′)	Reverse (5′-3′)
PI3K	AGTAGGCAACCGTGAAGAAAAG	GAGGTGAATTGAGGTCCCTAAGA
AKT	AGCGACGTGGCTATTGTGAAG	GCCATCATTCTTGAGGAGGAAGT
mTOR	GCAGATTTGCCAACTATCTTCGG	CAGCGGTAAAAGTGTCCCCTG
PTEN	TGGATTCGACTTAGACTTGACCT	GGTGGGTTATGGTCTTCAAAAGG
CCND1	GCTGCGAAGTGGAAACCATC	CCTCCTTCTGCACACATTTGAA
*β*-Actin	TGACGTGGACATCCGCAAAG	CTGGAAGGTGGACAGCGAGG

## Data Availability

The data that support the findings of this study are available from the corresponding author upon reasonable request.
